# Accelerative Effect of Cinnamon Nanoparticles as well as HAMLET on Healing of Wounds Infected with MRSA in Diabetic Rats

**DOI:** 10.1155/2021/9984540

**Published:** 2021-12-28

**Authors:** Ramezani Ali, Najafpour Alireza, Farahpour Mohammad Reza, Mohammadi Rahim

**Affiliations:** ^1^Department of Clinical Sciences, Faculty of Veterinary Medicine, Urmia Branch, Islamic Azad University, Urmia, Iran; ^2^Department of Surgery and Diagnostic Imaging, Faculty of Veterinary Medicine, Urmia University, Urmia, Iran

## Abstract

**Objective:**

The aim of the present study was to investigate the effect of cinnamon nanoparticles (CNPs) on healing of wounds infected with methicillin-resistant *Staphylococcus aurous* with human alpha-lactalbumin made lethal to tumor cells sensitization in diabetic rats.

**Methods:**

We included fifty diabetic male rats and divided them into 5 groups. There were 10 rats in each group as follows: CONTROL group: we did not infect the CONTROL group. The wound was only covered with sterile saline 0.9% solution (0.1 mL). INFCTD group: in this group, the wounds were infected with MRSA and covered with sterile saline 0.9% solution (0.1 mL). INFCTD-HMLT group: in this group, the wounds were infected with MRSA and HAMLET (100 *μ*g). INFCTD-CNM group: in this group, the wounds were infected with MRSA and 0.1 mL CNPs (1 mg/mL) were applied topically to wounds. INFCTD-HMLT-CNM group: in this group, the wounds were infected with MRSA, HAMLET (100 *μ*g), and 0.1 mL CNPs (1 mg/mL).

**Results:**

Bacteriology, wound area reduction measurements, biochemistry, histomorphometrical studies, hydroxyproline levels, and reverse transcription polymerase chain reaction for caspase-3, Bcl-2, and p53 showed significant difference between rats in the INFCTD-HMT-CNM group in comparison with other groups (*P* < 0.05).

**Conclusions:**

Accelerated healing of diabetic wounds infected with MRSA showed that local application of cinnamon nanoparticles along with HAMLET sensitization on *S. aureus*-infected wound could be taken into consideration.

## 1. Introduction

Diabetes mellitus, a metabolic disease, is a public issue which results in wounds in chronic form as a result of accumulation of anomalous blood glucose and results in neuropathy, arterial impairment, and disturbing function of numerous tissues and organs [1]. Lots of human beings are affected by diabetes, and it consumes bulky amount of medical expenses. Diabetic foot ulcer, a persistent infection, ensues due to poor circulation, imperfect nutrients, and inflammation. Antibiotics are used to manage diabetic wounds; however, the common serious issue is drug resistance. Hence, it is vital to design novel treatments to accelerate the diabetic wound healing process [2]. Precisely, a coordinated sequence of actions that are typically present in repair cannot be observed in diabetic wounds, and bacterial contamination additionally deteriorates the healing procedure. Innovative healing alternatives for the management of multidrug-resistant *Staphylococcus aureus* infections are immediately required. The occurrence of wound infections that result in amputation gets to more than fifty percent [3, 4].

Nosocomial infections are mainly caused by *S. aureus*. MRSA accounts for the most prevalent infections in skin [5]. It seems that multidrug-resistant *S. aureus* infections end up with a high rate of death with related massive expenses [6]. In spite of the high mortality rate, rather scarce new antibacterial agents are there in the medical system [7]. Furthermore, most of antibiotics produced in the recent years are molecules reengineered from the present antimicrobial groups [8]. Henceforth, innovative healing substitutions for the management of multidrug-resistant *S. aureus* infections are of high importance.

It has been demonstrated that human alpha-lactalbumin made lethal to tumor cells also bears bactericidal activities *in vitro*. It has been indicated that in *in vitro* and *in vivo* conditions, HAMLET as well as current antimicrobials worked against multidrug-resistant staphylococci [9, 10].

Nowadays, products from various fragments of the plants (aromatic types) have been widely applied for medical intentions [11]. Like nanomaterials of metallic origin, the nanoparticles of organic origins, natural herbs, are preferred because of the existence of activated agents with biocompatible properties that are abundant, easily stabilized, and safely handled [12]. *Cinnamomum cassia* (bearing polyphenol and cinnamaldehyde compounds) has been utilized extensively all over the world because of bearing healthy nutritious components. Irreplaceable qualities like safety, bioactivity, nontoxicity, and antimicrobial ability have made cinnamon compounds appropriate for various purposes [13].

Cinnamon nanoparticles (CNPs) were confirmed to be operational as antibacterial agents. The sensitivity of structure, morphology, and optical and antibacterial characteristics of CNPs to the variation of laser ablation energy have already been demonstrated. Systematic characterizations of the CNPs have demonstrated the practicability of monitoring their morphology in an appropriate method that is profitable for medical purposes [14, 15].

Polyphenol and cinnamaldehyde compounds in *Cinnamomum cassia* have been used worldwide as traditional herbal medicine and healthy nutrition element [14]. Unique attributes including safety, bioactivity, nontoxicity, and antibacterial efficacy make cinnamon compounds suitable for different applications; therefore, in-depth understanding of the antibacterial effectiveness of the bioactive components of cinnamon (extract or powder) may require an accurate synthesis method to produce CNPs with controlled morphology [14].

In order to investigate the healing effects of cinnamon nanoparticles on infected diabetic wounds in the presence of human alpha-lactalbumin made lethal to tumor cells, the present work was conducted to know whether CNPs could be able to improve and accelerate the wound healing process in an animal model.

## 2. Materials and Methods

### 2.1. Research Materials

Cinnamon sticks were purchased from a local supermarket (XXX, XXX). The specimen was identified by a botanist in the herbarium of the Faculty of Agriculture (deposition number 17339). In order to synthesize the CNPs, the ethanol of research grade (C_2_H_5_OH, 96%, Sigma-Aldrich) was utilized. We cut cinnamon sticks into small pieces (20 × 10 × 3 mm), and with an ultrasonic bath with acetone solvent, we cleaned them. Then, they were washed with purified water to remove contaminants.

### 2.2. Synthesis of CNPs

The nanoparticles of cinnamon dissolved in ethanol liquid medium were prepared via PLAL based on others [14]. First, the cinnamon stick as a target material was immersed at the 27 cm^3^ cubic container bottom with 5 ml liquid ethanol as growth solution. The laser irradiation “A Q-switched 1064-Nd: YAG laser (10 ns pulse duration, repetition rate 1 Hz, and varying laser energy 20-100 mJ) was directly focused on the surface of the target through a lens of focal length 80 mm. The distance between the laser lens and cinnamon surface target was positioned at 17 mm because of the refraction of the light phenomenon” was done as previously described [14]. Details of the methodology of preparation of the nanoparticles can be found in works of Salim et al. [14].

### 2.3. Analytical and Characterization Methods of CNPs

The characterization methods were performed based on the others [15]. Transmission electron microscopy (TEM), field emission scanning electron microscopy (FESEM), energy-dispersive X-ray spectroscopy (EDX), and X-ray photoelectron spectroscopy (XPS) were adopted to assess the morphology and topography of the samples as well as elemental chemical surface analysis. The size distribution of the nanoparticles was detected through a Zetasizer Nano ZS (Malvern Instruments Limited) particle analyzer. The FESEM instrument was used at an accelerating voltage at 10 kV. The synthesized CNPs were subjected to Fourier-transform infrared (FTIR; range 4000–400 cm^−1^) and photoluminescence (PL; range 200–800 nm) spectroscopy (UV-visible spectrophotometer, PerkinElmer, and Cary fluorescence spectrophotometer) to investigate the optical properties, functional groups, and structural defects. The X-ray diffraction (XRD) pattern of CNPs was recorded via a PANalytical PW3050/60 X-ray diffractometer equipped with Cu-K*α* radiation source (*λ* = 1.5406 Å) operated at 40 kV and 30 mA. An electron paramagnetic resonance (EPR) investigation on a Bruker ELEXSYS E500 X-band (~9.45 GHz) spectrometer was set to detect the paramagnetic defects in the structure as previously described [15].

### 2.4. Ethical Considerations

The Guide of the National Academy of Sciences published by the National Institutes of Health (NIH Publication No. 85-23, revised 1985) was followed in the present study. The Institutional Ethical Committee of the university approved the procedures in order to minimize any potential pain of the animals under ethical code IR.IAU.URMIA.REC.1400.023.

### 2.5. Preparation of HAMLET

We followed the methods of others to prepare the HAMLET [16]. In this method, ethylenediaminetetraacetic acid- (EDTA-) treated, partially unfolded *α*-lactalbumin as well as oleic acid (C18:1) on an anion exchange matrix was converted to a stable protein-lipid combination. The latter complex was again suspended in phosphate-buffered saline (pH = 7.4) in all formulations.

### 2.6. Induction of Diabetes and Monitoring the Blood Glucose Levels during the Study Period

We followed the methods of others to develop diabetes [16]. Accordingly, the rats underwent fasting for one night. Then, the animals received 60 mg/kg in 0.9% sterile saline of streptozotocin intraperitoneally. We approved hyperglycemia when the blood glucose level was 15 mmol/L or greater two days after streptozotocin administration using a glucometer (Ames Glucostix; Miles Laboratories). Three days after development of diabetes, we created wounds on the dorsum of the animals. Levels of blood glucose in the animals within the study period were acquired to ensure that the animals were diabetic throughout the study period (Table 1).

### 2.7. The Wound Creation Procedures and Infection Induction

We followed the methods of others to develop wounds and infection [16]. To anesthetize the animals, they received combination of 70 mg/kg ketamine and 5 mg/kg xylazine intraperitoneally. Following surgical preparation of the dorsum of the animals, we created a wound in a circular fashion 10 mm in diameter. We dressed the wound using a small gauze, and afterward via intradermal injection, the wound was inoculated with 5 × 10^7^ colony-forming units (CFU) of MRSA (commercially available as *S. aureus* ATCC 43300). We returned back the animals to their cages and keep them monitored for 24 hours.

### 2.8. Randomization and Grouping of Animals

We followed the methods of others for randomization and grouping of animals [1]. We randomized fifty diabetic male rats into 5 groups. There were 5 rats in each group as follows:

1. CONTROL group: we did not infect the CONTROL group. The wound was only covered with sterile saline 0.9% solution (0.1 mL)
2. INFCTD group: in this group, the wounds were infected with MRSA and covered with sterile saline 0.9% solution (0.1 mL)
3. INFCTD-HMLT group: in this group, the wounds were infected with MRSA and HAMLET (100 *μ*g)
4. INFCTD-CNM group: in this group, the wounds were infected with MRSA and 0.1 mL CNPs (1 mg/mL) were applied topically to wounds
5. INFCTD-HMLT-CNM group: in this group, the wounds were infected with MRSA, HAMLET (100 *μ*g), and 0.1 mL CNPs (1 mg/mL)

We continued the use of test solutions for 10 days and each day for two times. Animal housing was in standard conditions of temperature (22 ± 3°C), humidity (60 ± 5%), and a 12-hour light/dark cycle. They were fed standard pellet diet and tap water. The animals were carefully monitored for any possible systemic infection. In the case of infection, the affected animals were excluded from the experiment and replaced by another one using the corresponding protocol.

### 2.9. Microbiological Tests

We followed the methods of others for microbiological tests [16]. We aseptically excised the granulated tissues 7 and 14 days after wound creation to get the total bacterial count. To do this, we crushed and homogenized 0.1 g of tissue specimen in a sterile mortar with 10 mL of sterile saline. To get the final concentration of 10^−5^, we serially diluted the prepared specimen in a tube with 9 mL of sterile saline. We cultured the diluted samples superficially and duplicated them on plate count agar (Merck KGaA) and incubated them at 37°C for 48 hours. We counted all colonies after incubation, and results were presented as CFU/g of granulation tissue.

### 2.10. Planimetric Studies in the Excisional Wound Model

We followed the methods of others for planimetric studies in the excisional wound model [16]. In brief, the process of healing was investigated via measurement of reduction in the wound surface; therefore, we put a ruler as a scale next to the wounds, and with a digital camera immediately after wounding and on days 6, 9, 12, 15, 18, and 21, photographs were taken. We used the Measuring Tool of Adobe Acrobat 9 Pro Extended software (Adobe Systems Inc.) to measure the wound area.

### 2.11. Biochemical Investigations

We followed the methods of others for biochemical investigations [16, 17]. To do this, we took the specimens of wound tissue and assessed their enzyme activities. We used a mortar to grind the samples. We treated one-half gram of each sample with 4.5 mL of an appropriate buffer. Ultra-Turrax homogenizer (IKA Werke) mixture was used to homogenize the samples. Following filtration of the homogenates with the use of a refrigerator centrifuge, the samples were centrifuged at 4°C. For assessments of the enzymatic activities at room temperature, supernatants were used. The activity of the following biochemical parameters was assessed:

- Superoxide dismutase (SOD)
- Total nitric oxide synthase (tNOS)
- Malondialdehyde (MDA)
- Myeloperoxidase (MPO)
- Total glutathione (tGSH)
- Glutathione peroxidase (GPO)
- Glutathione reductase (GSHRd)
- Glutathione S-transferase (GST) analyses
- Isolation of DNA from tissue
- cDNA hydrolysis with formic acid measurement of 8-hydroxy-2′-deoxyguanosine (8-OH Gua)

### 2.12. Histological Preparation and Quantitative Morphometric Studies

After wound creation, on days 7, 14, and 21, a tissue sample from the edge of the wound as well as normal skin was taken and fixated in an appropriate fixative (10% buffered formalin). The samples underwent routine tissue processing of dehydration and paraffin wax embedding. 5 *μ*m sections were stained with hematoxylin and eosin (H&E) and Masson's trichrome stains. Using light microscopy, photomicrographs of various stages of the healing processes were scrutinized. Mononuclear cells, polymorphonuclear cells, and fibroblastic aggregation were quantitatively analyzed. Image analyzing software (Image-Pro Express, version 6.0.0.319, Media Cybernetics) was adopted to score morphological results. Using a five-step scoring system, the histological parameters were classified based on the intensity of occurrence (−, absence; +, discrete; ++, moderate; +++, intense; and ++++, very intense) [16, 17].

### 2.13. Immunohistochemical Staining for Angiogenesis

As previously described [16] for immunohistochemical (IHC) staining, the following steps were followed: first, in a hot air oven (Venticell, MMM Einrichtungen), the sectioned samples were heated for about 25 min at 60°C. Then, using xylene and alcohol gradient, the sections were dewaxed and rehydrated, respectively. For retrieval of antigen, 10 mM sodium citrate buffer was used. Based on the manufacturer's instructions (Biocare), IHC staining was performed.

To block endogenous peroxidase, we used peroxidase blocking solution. The samples were incubated with CD31 (Biocare) biotinylated primary antibodies (rabbit/anti-mouse, 1 : 500) for 15 min after washing with a buffer. The samples were put in a buffer bath after rinsing with a buffer. The samples were incubated for 15 min after putting in a chamber with sufficient humidity with streptavidin-HRP and then were washed with a buffer and put in a buffer bath. The sections were then treated with a DAB (3,3′-diaminobenzidine) chromogen and following rinsing as well as counterstaining with hematoxylin (for 5 sec) were incubated for 5 minutes. For dipping the samples, a weak ammonia (0.037 M) was used. After rinsing with distilled water, they were placed on a coverslip and observed under a light microscope.

### 2.14. Hydroxyproline Level Investigations

We followed the methods of others to measure contents of hydroxyproline in the tissue [17]. To dry the harvested tissues to constant weight, a hot air oven at 60 to 70°C was used. Then, the sample was hydrolyzed in 6 N HCl at 130°C for 4 hours. To neutralize the hydrolysate to pH 7.0, chloramine-T oxidation was applied for 20 minutes. We added 0.4 M perchloric acid to stop the reaction. Using the Ehrlich reagent at 60°C, a color was established. Then, an ultraviolet-visible spectrophotometer (CamSpec M330) at 557 nm was used.

### 2.15. RNA Isolation and cDNA Synthesis

As previously described [16], we extracted total RNA from samples of tissues of experimented rats. The standard TRIzol method was adopted for extraction. We homogenized 50 to 100 mg of samples in 1 mL of TRIzol. To prevent contamination of genomic DNA, carefully the colorless aqueous phase was collected. We isolated RNA, determined it spectrophotometrically (260 nm and 260/280 = 1.8-2.0), and stored it at −70°C. Based on what the manufacturer (Fermentas GmbH) instructed, to perform RT-PCR, cDNA was produced in a 20 *μ*L reaction mixture with 1 *μ*g RNA, oligo (dT) primer (1 *μ*L), 5× reaction buffer (4 *μ*L), RNAse inhibitor (1 *μ*L), 10 mM dNTP mix (2 *μ*L), and M-MuLV Reverse Transcriptase (1 *μ*L). The cycling procedure for 20 *μ*L reaction mix was 5 min at 65°C, followed by 60 min at 42°C and 5 min at 70°C to terminate the reaction.

### 2.16. RT-PCR for Caspase-3, Bcl-2, and p53

As previously described [16], we performed PCR reaction (with volume of 25 *μ*L) with the PCR master mix of volume 12.5 *μ*L, forward and reverse specific primers (each of 0.75 *μ*L), and cDNA as a template (1 *μ*L) and nuclease-free water (10 *μ*L). We did PCR in the following steps: first—general denaturation: at 95°C for 3 minutes, 1 cycle, followed by 40 cycles of 95°C for 20 seconds; second—annealing temperature: 62°C for Bcl-2, 52°C for p53, and 50°C for caspase-3 for 60 seconds; and third—elongation: -72°C for 1 min and 72°C for 5 min.

The products of reaction were isolated using 1.5% agarose gel. They were visualized using ethidium bromide staining with Gel Doc 2000 (Bio-Rad). The forward and reverse primers of caspase-3, Bcl-2, and p53 are depicted in Table 2.

### 2.17. Statistical Analysis

Kruskal-Wallis variance analysis was adopted for differences among groups. Where the *P* value (from the Kruskal-Wallis test statistics) was statistically significant, multiple comparison tests were utilized to get the differences. The Mann-Whitney *U* test was used for comparison among days. For retrieving possible multiple comparisons, the Bonferroni correction was utilized. We utilized SPSS 11.5 (SPSS Inc.) for the analyses and considered the *P* value < 0.05 as the significant level.

## 3. Results

### 3.1. Analytical Assessments

#### 3.1.1. Microstructural Characterization

The TEM image of CNPs (Figure 1(a)) evidently illustrates that the particles were typically sphere-shaped with a size range of 10 to100 nm (zeta potential: -50.0 mV and polydispersity index: 0.484). The even dispersion and nearly sphere-shaped CNPs could be detected in the FESEM image (Figure 1(b)). The mean value for sizes of the NPs was about 43 ± 17 nm based on the dynamic light scattering (DLS) technique (Figures 1(c) and 1(d)).

#### 3.1.2. Physicochemical Characterization

Figure 2(a) illustrates the XRD pattern of the synthesized CNPs. The well-defined quite broad peaks with a high-intensity pattern indicated the production of the nanoparticle phase. There were no additional peaks in the resolution limit of the X-ray diffractometer indicating synthesis of CNPs.  Figure 2(b) shows the produced CNPs demonstrated by EDX. The EDX spectrum confirmed purity of produced CNPs. The EPR curve analysis was according to the calculated *g*-values from a spectrum formed of a symmetrical Lorentzian shape (Figure 3(a)). The synthesized CNPs were examined by analysis of the surface of XPS as well (Figure 3(b)) indicating a complete survey scan, and peaks were attributed to the CNPs. The results of FTIR indicated no significant difference between particles of nanocinnamon (Figure 4(a)) and cinnamon (Figure 4(b)).

### 3.2. Microbiological Examinations and Healing Rate Reduction in the Wound Area

Significantly lower numbers of *S. aureus* inoculated in the wounds were observed in the INFCTD-HMLT-CNM group compared to INFCTD-HMLT and INFCTD-CNM groups (*P* < 0.05). None of animals died due to infection or anesthesia. In the CONTROL group, colonies of *S. aureus* were not observed. Application of CNPs and HAMLET significantly diminished the rate of total bacterial count in the INFCTD-HMLT-CNM group compared to INFCTD-HMLT and INFCTD-CNM groups following days 7 and 14 after wounding (*P* < 0.05; Table 3).  Table 4 shows values of percentage of contraction of wound in experimental animals throughout the experiment. The rate of healing of wounds in the INFCTD-HMLT-CNM group was significantly higher than those of INFCTD-HMLT and INFCTD-CNM groups (Figure 5) (*P* < 0.05).

### 3.3. Biochemical Findings

Topical usage of cinnamon nanoparticles resulted in significant augmentation in the activity of SOD in the INFCTD-HMLT-CNM group in comparison with activity of SOD in other groups (*P* < 0.05). The activity of tNOS was declined in INFCTD-HMLT-CNM animals with a significant decrease compared to other groups (*P* < 0.05). Cinnamon nanoparticles significantly diminished MDA level in the INFCTD-HMLT-CNM group in comparison with other experimental groups (*P* < 0.05). The cinnamon nanoparticles resulted in significant diminution level of MPO in tissues of INFCTD-HMLT-CNM animals (*P* < 0.05). Levels of GSH, GPO, GSHRd, and GST in INFCTD-HMLT-CNM animals were significantly increased in comparison with other experimental groups (*P* < 0.05). Significant decrease was found in the levels of 8-OHGual/Gua, a DNA damage product, in the INFCTD-HMLT-CNM group in comparison with other experimental groups (*P* < 0.05, Figure 6).

### 3.4. Histological and Morphometric Findings

Significant differences between INFCTD-HMLT-CNM and other experimental groups were found regarding reepithelialization, new vessel formation, acute hemorrhage, congestion, cellular infiltration, collagen production, and edema. In the present study, significantly higher scores were observed in reepithelialization and new vessel formation in INFCTD-HMLT-CNM group rats compared to INFCTD-HMLT and INFCTD-CNM groups (*P* < 0.05). Mean values for the cell count and also mean rank of the qualitative study of the wound score in INFCTD-HMLT-CNM animals were significantly higher than those of INFCTD-HMLT and INFCTD-CNM animals (*P* < 0.05; Table 5 and Figures 7–10).

### 3.5. Results of Immunohistochemistry for New Vessel Formation

Analyses of immunohistochemistry demonstrated that utilization of cinnamon nanoparticles as well as HAMLET significantly augmented the angiogenesis (*P* < 0.05; Figure 11).

### 3.6. Hydroxyproline Content of Wound

The results of our investigation showed that hydroxyproline contents in the CONTROL, INFCTD, INFCTD-HMLT, INFCTD-CNM, and INFCTD-HMLT-CNM groups were 47.54 ± 3.54, 67.51 ± 4.15, 65.76 ± 5.71, 73.89 ± 5.37, and 97.11 ± 3.73 mg/g, respectively. Hydroxyproline levels were significantly augmented in the INFCTD-HMLT-CNM animals indicating deposition of additional collagen in comparison with INFCTD-HMLT and INFCTD-CNM groups (*P* < 0.05).

### 3.7. RT-PCR Results for Caspase-3, Bcl-2, and p53

The levels of mRNA of caspase-3, Bcl-2, and p53 genes were analyzed to assess the ratio of proliferation of cells on day 8 postwounding. The findings indicated that the application of cinnamon nanoparticles as well as HAMLET ended up with a significant rise at the mRNA level of caspase-3 in comparison with other animals (*P* < 0.05) (Figure 12).

## 4. Discussion

Infection potentiates dysfunction of wound healing in diabetes and results in extensive amount of morbidity and mortality all over the world [18].

Deficiency in signaling of cells and molecules that are required for the regular process in wound healing like neovascularization, generation of granulation tissue, epithelialization, and tissue remodeling occurs in diabetic patients and results in the impairment of wound healing in diabetes.

The regular repair process occurs in healthy patients at an optimum degree; however, in diabetic individuals, it is commonly delayed or even totally compromised [19]. The process of wound repair in diabetic individuals is compromised and delayed as a result of increase in blood glucose levels. Increased glucose of blood inhibits cell proliferation and diminishes collagen formation that leads to reduced chemotaxis and phagocytosis [20]. Raised levels of blood glucose, decreased growth factor levels, and inhibited fibroblast proliferation have been demonstrated to compromise wound healing [20]. The wound repair process occurs spontaneously without further help; however, numerous risk factors such as diseases, infection, blood supply, and nutritional status may deteriorate the normal process [21].

MRSA infections are growing and becoming a severe hazard in the hospitals and the public. Common antibiotic resistance makes managing MRSA infections expensive and problematic. Contraction of wound and subsequent reduction in the area of wound, a chief end point in our investigation, were hastened by treating the MRSA-infected diabetic wounds with the topical use of cinnamon nanoparticles as well as HAMLET. In our study, the existence of necrotic tissue, clotting, crust, epithelialization, formation of granulation tissue, and microbial number were affected demonstrating that cinnamon nanoparticles as well as HAMLET could combat MRSA infections. The local use of HAMLET in the site of the wound resulted in noteworthy activity in wound repair signifying that it has resulted in MRSA eradication.

A substantial reduction in the wound area was observed in the excisional wound model. This showed enhanced maturation of collagen by increase in cross-linking. The equilibrium between production and degradation and collagen deposition is crucial in wound repair and improvement of strength of wound [22]. Hydroxyproline, a chief constituent of the collagen, allows the collagen helix sharp twisting. It supports firmness to unique structure of collagen via hydrogen bond formation. Hydroxyproline is rarely located in proteins other than collagen, and that is why quantity of hydroxyproline has been considered a scale to approximate content of collagen [23]. Increase in quantity of hydroxyproline in the INFCTD-HMLT-CNM group specified increase in collagen quantity because it is a straight estimation of collagen production. Nanoparticles of cinnamon have been shown to signify a novel local antibacterial and wound healing adjuvant for cutaneous damage and infected burn wounds [24]. Our findings revealed that cinnamon nanoparticles as well as HAMLET considerably decreased tissue bacterial count and promoted the repair phases in infected diabetic wounds. Hence, INFCTD-HMLT-CNM animals revealed condensed phases of inflammation and homeostasis and increased phases of proliferation and maturation. Regarding the significance of the bacterial infection and existence of pathogens in wound, counting the colonies of MRSA in the area of wound was performed in the present study. The findings revealed that the infection was managed after topical use of cinnamon nanoparticles as well as HAMLET. Inflammation is a leading pace to remove tissue cellular debris along with effective response to microbial infection [25, 26]. Accordingly, quick response is required to manage the inflammation. Within inflammatory phase neutrophils, macrophages and lymphocytes penetrate to the injury site [26, 27]. Analyses of light microscopy indicated that in the INFCTD-HMLT-CNM group, infiltration of mononuclear immune cell was significantly increased eight days after wound creation. This condition is crucial in removing the infection and accelerating the repair course via the significant role of inflammatory cells, particularly macrophages, and establishing the granulation tissue. Hence, the antibacterial characteristic of nanoparticles of cinnamon as well as HAMLET could be mainly associated with these elements. The findings of our study revealed that nanoparticles of cinnamon as well as HAMLET resulted in enhanced proliferation of cells and that distribution of fibroblasts and fibrocytes in 1 mm^2^ of the wound area was considerably higher compared to other groups. Considering the crucial role of fibroblasts and fibrocytes in the formation of collagen [26], it was concluded that raised deposition in collagen in the INFCTD-HMLT-CNM group was associated with high cellularity of fibroblasts and fibrocytes. Increase in new vessel formation eight days after wound creation revealed that nanoparticles of cinnamon as well as HAMLET could accelerate the repair process by inducing infiltration of cells.

Within the inflammatory stage, numerous radicals are produced as a result of damage [28]. Radicals are frequently connected to oxidative stress, which result in peroxidation of lipid and compromised wound repair [28]. Decrease in oxidative stress increases the inflammatory reaction, and our results revealed that cinnamon nanoparticles could be able to remove radicals [29].Therefore, in the present study, the biochemical indices were significantly improved in INFCTD-HMLT-CNM animals in comparison with those of other experimental groups. The results of histochemistry in the present study for dispersion of vessels were consistent with these findings. INFCTD-HMLT-CNM animals showed significantly higher new vessel formation in comparison with INFCTD-CNM and INFCTD-HAMLET groups. Enhanced new vessel formation after wound creation indicated that cinnamon nanoparticles as well as HAMLET could promote the healing process due to enhancement in cellular infiltration [17].

The crucial fact to inflammation termination is the activity of apoptosis in the immune cells [30]. The mediators that promote infiltration of activated immune cells into inflammation help defend the tissue in contradiction of infection in the inflammation response. At termination of the inflammation, apoptosis of the immune cells occurs and macrophages clear the apoptotic cells. The removal of apoptotic cells by macrophages is correlated with termination of wound inflammation and onset of active tissue formation in wound [31].

In the family of proteins, the Bcl-2 inhibits apoptosis as apoptosis pathway effectors [32, 33]. However, the guardian of the genome, caspase and p53, regulates the destiny of damaged cells via detection and ending the cell cycle. In damaged tissue, increase in the levels of p53 and caspase is observed to trigger apoptotic activity of the immune cells that results in the exclusion of the immune cells. Following this phase, the Bcl-2 inhibits the apoptotic activity that induces the proliferation of cells [34]. In the present study, analyses of RT-PCR indicated that in INFCTD-HMLT-CNM animals, expressions of caspase 3, Bcl-2, and p43 were amplified. Therefore, it might be estimated that nanoparticles of cinnamon as well as HAMLET improved the proliferation of the cells via upregulation in the expression of caspase 3, Bcl-2, and p43. Sensitization of the bacterial pathogens to traditional antimicrobial agents has already been demonstrated by HAMLET [35–39].

## 5. Conclusions

The aim of the present work was to indicate that cinnamon nanoparticles as well as HAMLET could display antibacterial activity in contradiction of MRSA. This was the first record of the literature on the effectiveness of cinnamon nanoparticles as well as HMLET in the improvement of MRSA-infected diabetic wounds. Hence, our results demonstrated that HAMLET could make cinnamon nanoparticles valuable for the management of wounds infected with MRSA and could offer potential to pay more attention to this harmless and easily available agent to be topically applied in wounds with infection in diabetes. Studies in a dose-response manner are required to assess different concentrations for the cinnamon nanoparticles as well as HAMLET to determine optimal dosages to accomplish extreme efficacy.

## Figures and Tables

**Figure 1:** (a) TEM and (b) FESEM images of the synthesized CNPs. Size distribution of the nanoparticles according to the (c) number and (d) volume by dynamic light scattering.

**Figure 2:** (a) Pattern of diffraction of X-ray and (b) spectrum of EDX spectroscopy of the produced CNPs.

**Figure 3:** (a) The EPR analysis curve according to the measured *g*-values from a spectrum formed of a symmetrical Lorentzian shape. (b) Spectrum of X-ray photoelectron spectroscopy of the synthesized CNPs.

**Figure 4:** Spectrum of Fourier-transform infrared spectrophotometry (a) of CNPs and (b) cinnamon particles.

**Figure 5:** Serial photographs of wounds on different days in experimental groups: (a) CONTROL, (b) INFCTD, (c) INFCTD-HMLT, (d) INFCTD-CNM, and (e) INFCTD-HMLT-CNM.

**Figure 6:** Bar graph shows comparison of the activities of biochemical parameters and a DNA damage product of 8-OHGual/Gua in the experimental groups. Results were presented as mean ± SEM. ^∗^*P* < 0.05 versus INFCTD, INFCTD-HMLT-CNM, and INFCTD-HMLT groups. SOD: superoxide dismutase; tNOS: total nitric oxide synthase; MDA: malondialdehyde; MPO: myeloperoxidase; tGSH: total glutathione; GPO: glutathione peroxidase; GSHRd: glutathione reductase; GST: glutathione S-transferase; 8-OHGual/Gua: 8-hydroxy-2-deoxyguanosine.

**Figure 7:** The graph shows the number of polymorphonuclear cells (PMN) in the excisional model of the animals in the experimental groups. Results were presented as mean ± SEM. ^∗^*P* < 0.05 versus INFCTD, INFCTD-HMLT-CNM, and INFCTD-HMLT groups.

**Figure 8:** Bar graph shows the number of mononuclear cells (MNC) in the excisional model of the animals in the experimental groups. Results were expressed as mean ± SEM. ^∗^*P* < 0.05 versus INFCTD, INFCTD-HMLT-CNM, and INFCTD-HMLT groups.

**Figure 9:** Bar graph shows the number of fibroblasts in the excisional model of the animals in the experimental groups. Results were expressed as mean ± SEM. ^∗^*P* < 0.05 versus INFCTD, INFCTD-HMLT-CNM, and INFCTD-HMLT groups.

**Figure 10:** Histomorphometrical analyses 14 days following the creation of wounds in the excisional wound model: (a) CONTROL, (b) INFCTD, (c) INFCTD-HMLT, (d) INFCTD-CNM, and (e) INFCTD-HMLT-CNM. Wounds with the surrounding skin were prepared for histological microscopic evaluation by hematoxylin and eosin staining. Scale bar: 60 *μ*m.

**Figure 11:** Immunohistochemical staining for CD31 on day 14 postwound creation: (a) CONTROL, (b) INFCTD, (c) INFCTD-HMLT, (d) INFCTD-CNM, and (e) INFCTD-HMLT-CNM. Scale bar: 50 *μ*m.

**Figure 12:** Reverse transcription polymerase chain reaction results for mRNA levels of Bcl-2, caspase-3, and p53 based on *β*-actin intensity. Cinnamon nanoparticles as well as HAMLET increased the mRNA level of caspase-3, Bcl-2, and p53 on day 7 postoperation. All data are presented as mean ± SEM. ^∗^*P* < 0.05 versus INFCTD, INFCTD-HMLT-CNM, and INFCTD-HMLT groups: (A) CONTROL, (B) INFCTD, (C) INFCTD-HMLT, (D) INFCTD-CNM, and (E) INFCTD-HMLT-CNM.

**Table 1:** Blood glucose levels (mg/dL) of the animals within the experiment days. Data are expressed as mean ± SD.

Groups	Day of injection^∗^	2 days postoperation	7 days postoperation	14 days postoperation	21 days postoperation
CONTROL	81.7 ± 9.2	363.4 ± 21.5	277.3 ± 23.4	233.7 ± 20.4	227.7 ± 20.9
INFCTD	79.5 ± 8.0	361.7 ± 22.8	270.5 ± 21.5	230.3 ± 21.8	225.3 ± 22.7
INFCTD-HMLT	81.7 ± 9.3	360.4 ± 21.5	274.7 ± 23.7	234.7 ± 20.4	227.7 ± 20.3
INFCTD-CNM	79.7 ± 9.5	363.7 ± 21.7	271.8 ± 20.5	231.3 ± 22.6	225.3 ± 21.6
INFCTD-HMLT-CNM	80.4 ± 9.0	362.3 ± 22.5	275.6 ± 20.7	233.7 ± 21.9	225.3 ± 21.5

^∗^“Day of injection” was three days before operation, and it denotes the day when the streptozotocin was injected for the induction of diabetes.

**Table 2:** Sequences of the primer pairs and product sizes used for RT-PCR.

Gene name	Forward	Reverse	Product size
Caspase-3	5′-TACCCTGAAATGGGCTTGTGT-3′	5′-GTTAACACGAGTGAGGATGTG-3′	446 bp
Bcl-2	5′-CGCCCGCTGTGCACCGAGA-3′	5′-CACAATCCTCCCCCAGTTCACC-3′	228 bp
P53	5′-GAGGAGATGATGCTGCTGAG-3′	5′-TGCTGCTGCTGCTATTACC-3′	250 bp

**Table 3:** Wound bacterial count in experimental groups on two time points (day 7 and day 14 postinfection).

Groups	Wound granulation tissue bacterial count (CFU/g)	
	On day 7	On day 14
CONTROL	0.00 ± 0.00	0.00 ± 0.00
INFCTD	1371.76 ± 281.62	1227.59 ± 238.74
INFCTD-HMLT	1388.59 ± 217.59	982.88 ± 226.23
INFCTD-CNM	1215.48 ± 248.69	942.32 ± 247.76
INFCTD-HMLT-CNM	531.19 ± 78.19^∗^	257.36 ± 65.32^∗^

CFU: colony-forming units; MRSA: methicillin-resistant *Staphylococcus aureus*; HAMLET: human *α*-lactalbumin made lethal to tumor cells. ^∗^*P* < 0.05 versus INFCTD-HMLT and INFCTD-CNM groups.

**Table 4:** Impact of application of cinnamon nanoparticles as well as HAMLET on the circular excision wound contraction area (mm^2^). Values are given as mean ± SEM.

Wound area (mm^2^)						
Groups	Day 6	Day 9	Day 12	Day 15	Day 18	Day 21
CONTROL	251.53 ± 4.76	105.35 ± 5.18	88.74 ± 3.69	48.75 ± 3.35	27.28 ± 2.54	6.11 ± 2.10
INFCTD	261.45 ± 4.52	203.70 ± 4.45	185.17 ± 3.23	146.77 ± 3.93	98.68 ± 3.70	76.15 ± 3.87
INFCTD-HMLT	249.23 ± 4.43	206.74 ± 4.65	183.54 ± 9.67	147.50 ± 7.15	89.76 ± 2.55	74.38 ± 2.82
INFCTD-CNM	229.34 ± 4.76	195.56 ± 4.76	163.65 ± 3.63	103.70 ± 3.65	62.10 ± 3.15	42.66 ± 2.24
INFCTD-HMLT-CNM	111.23 ± 3.90^∗^	72.17 ± 2.76^∗^	33.72 ± 2.65^∗^	14.25 ± 1.76^∗^	4.88 ± 3.73^∗^	0.00 ± 0.00^∗^

The treated groups are compared by the Student *t*-test with other groups. ^∗^*P* < 0.05 versus INFCTD-HMLT and INFCTD-CNM groups.

**Table 5:** The histological parameters classified based on the intensity of occurrence in 5 levels described by others [17].

Histological parameter	Groups and days														
	CONTROL			INFCTD			INFCTD-HMLT			INFCTD-CNM			INFCTD-HMLT-CNM		
	7	14	21	7	14	21	7	14	21	7	14	21	7	14	21
Acute hemorrhage	+++	++	−	++++	+++	++	++++	+++	++	+++	+	+	+^∗^	−	−
Congestion	++++	+	−	++++	+++	++	++++	++	++	+++	+	+	+^∗^	−	−
Vascularization	+	++	+++	−	+	+	−	+	+	−	+	+++	+++^∗^	++++^∗^	++++^∗^
Epithelialization	−	+	++	−	+	+	−	+	+	+	++	+++	++^∗^	+++^∗^	++++^∗^
Collagen	+	++	++	−	+	+	−	+	+	+	++	+++	++^∗^	+++^∗^	++++^∗^

Classification of histological parameters according to the intensity of occurrence: − absence; + discrete; ++ moderate; +++ intense; and ++++ very intense. Histopathological damage was assessed as explained under Materials and Methods on days 7, 14, and 21 of the lesion. ^∗^*P* < 0.05 vs. INFCTD-HMLT and INFCTD-CNM groups.

## Data Availability

The data used to support the findings of this study are available from the corresponding author upon request.
